RETRACTED

# Prevention and Nursing Research of PICC Catheter-Related Complications in Patients with Digestive System Malignant Tumor Based on Smart Medical Block Chain

**DOI:** 10.1155/2021/5519722

**Published:** 2021-04-12

**Authors:** Ruxian Huang, Yan Jiang, Xiaoyun Le

**Affiliations:** Gastrointestinal Surgery, The Central Hospital of Wuhan, Tongji Medical College Huazhong University of Science and Technology, Wuhan 430000, Hubei, China

## Abstract

Malignant tumors of digestive system mainly include gastric cancer, colorectal cancer, and esophageal cancer, which generally need chemotherapy. PICC refers to peripherally inserted central venous catheter, which plays an important role in the treatment of malignant tumor patients with chemotherapy, and it has the characteristics of high success rate of puncture and reducing the pain of patients. Its principle is to use PICC catheter for drug delivery, which can effectively reduce the pain of tumor patients for multiple puncture, and also can avoid drug extravasation or local stimulation of drugs. However, PICC catheter-related complications cannot be ignored, to some extent, directly affect the treatment effect of patients, and increase the pain and burden of patients. Therefore, this paper proposes a study of PICC catheter-related complications and protective nursing for patients with digestive system cancer based on smart medical block chain. First of all, using the method of literature, this paper deeply studied the combination of smart medicine and block chain and further strengthened the research on PICC catheter-related complications. Based on this, we designed a study on the prevention and nursing of PICC catheter-related complications in patients with digestive system cancer. Before the implementation of nursing, the incidence of complications in patients with digestive system cancer was 17.35%; after the implementation of nursing, the incidence of complications decreased to 4.08%. The purpose of this study is to analyze the causes through clinical research and put forward the protective nursing measures of related diseases, so as to reduce the incidence of PICC-related complications.

## 1. Introduction

In recent years, many countries actively promote the development of large-scale medical data [1]. It is not only traditional medical institutions that promote medical information. At the same time, many pharmaceutical companies are also using big data to save high R&D costs. The medical industry is becoming one of the first traditional industries to enter the era of big data [2].

There is a lot of imagination space for smart medicine, but it is still a long way from reality. For now, the data information between domestic medical institutions does not flow and remains a serious problem [3], “islands of information” and the unequal distribution of medical resources are still a problem faced by medical wisdom, and, at the same time, privacy, security of medical data, and problems such as reliability have yet to be solved.

RETRACTED

Background: the choice of peripherally inserted central catheter (PICC) arm is usually decided by PICC nurses. Objective: to investigate the effect of arm type selection (dominant or nondominant) on the incidence of catheter-related complications and comfort in patients with PICCs. Design: cross sectional study. Methods: questionnaire and scale were used to investigate the general situation, catheter-related complications and comfort of 255 patients. They were divided into dominant arm group and nondominant arm group. Results: the obstruction rate and bleeding rate of PICC insertion site in nondominant group were significantly lower than those in the dominant group (*χ* = 9.829, *P* < 0.05; *χ* = 6.502, *P* < 0.05). The comfort degree of nondominant group was higher (*z* = 10.166, *P* < 0.01). Conclusion: nondominant arm insertion is associated with low incidence of catheter-related complications and high comfort of patients. Impact statement: these findings provide practical basis for nurses to make better choices. However, its defect is that it only considers the influence of arm shape and ignores the influence of many other factors [4]. Flores Moreno *m* background: in pediatrics, the incidence of peripherally inserted central catheter (PICC) complications is 30%–40%. The most common risk factors are the age of patients and the location of PICC. The purpose of this study was to describe the characteristics of PICCs and to identify the factors associated with withdrawal from PICCs due to complications. Methods: prospective cohort study. The patients ranged from 2 months to 18 years of age and were followed up until the withdrawal of PICC. Age, gender, medication, PICC location, caliber, number of lumens, days of PICC in patients, and the reasons for drug withdrawal were recorded. Univariate and multivariate analysis were performed. Results: a total of 225 patients were included. 33.02% of them withdrew from PICC due to complications. In bivariate analysis, age and location were associated with complications. Cox proportional hazard model was used [5]. Many factors of children are far different from those of adults in PICC operation, so it is of little reference significance for adults in PICC operation [6]. As people grow older and devote themselves to life, many people give up their commitment to things, which become their daily life. Many patients forget to receive treatment on time, while some patients do not receive treatment as planned, which reduces the efficiency of treatment. In some cases, the way in which nurses who care for the elderly and children remind patients of their schedules is not considered a successful solution because it depends on another person who may ignore or forget the exact time. With the popularity of smart phones [7], a technical solution is needed to help patients accurately determine the medication schedule and make them better control their medication. This paper presents an application running on iPhone, which is connected with smart drawer through Arduino board. The main purpose of this application is to organize and remind patients to take medicine on time. Drawers can be opened and closed through applications. Intelligent medicine has brought convenience to people, but we need to pay attention to relying on intelligent medical blindly and ignoring the physical and mental health of the elderly, especially mental health [8].

RETRACTED

The innovation of this paper lies in (1) the combination of qualitative analysis and quantitative analysis, fully based on the analysis of data, qualitative analysis; (2) the combination of theoretical research and empirical research, in-depth study of smart medical block chain technology and other theoretical bases, combined with the specific situation of patients with digestive system cancer, empirical research. (3) On the basis of smart medicine, we should make full use of the protective nursing method to reduce the incidence of PICC catheter-related complications and reduce the medical pain of patients with digestive system cancer.

## 2. PICC Catheter-Related Complications and Protective Care Research Methods in Patients with Malignant Tumors of the Digestive System Based on the Wisdom of the Medical Block Chain

### 2.1. Smart Medical

The future development of smart medicine is human's desire for health. The basic idea of intelligent medicine is “people-centered” [9]. The needs of patients can be solved by intelligent medicine. From entering the whole process of hospital service, we need the humanization of intelligent medicine. Intelligent medicine, especially in the service after treatment, can solve the shortcomings of interpersonal communication. Similarly, the needs of healthy people can also be solved through intelligent treatment. For example, from prevention to before the occurrence of diseases, we can find ways to eliminate the threat to subhealth status and then maintain health [10].

In fact, smart medicine is mainly composed of three main systems. The first is the hospital's intelligent service system [11]. Changes in the organizational structure of the hospital will bring changes to the staff of the hospital. They need to be socialized and have the ability to operate intelligently, such as intelligent device maintenance. The second is the regional health system [12]. The hospital is equipped with a reliable intelligent diagnosis system, which is comparable to the intelligence of most doctors and can achieve a more consistent way of thinking. High level doctors using the Internet for diagnosis and guidance, especially in the case of providing medicine, can change the current basic medical diagnosis in rural areas. The third is the personal health system [13]. Personal health system has more machines and products, especially intelligent nursing equipment. It has high commercial value. Although the current price of personal health equipment is extremely expensive, it will be able to achieve universal application in the future.

RETRACTED

The problem of intelligent medicine can be summarized into three main points. (1) The integration of information and data: the medical industry contains many aspects of information, including not only medicine, patient information, and equipment information, but also various diseases and treatment methods, which need technology to classify and sort them out [14]. (2) Data sharing and use: at present, a number of medical institutions and hospitals in China are in the state of data independence, without complete data sharing, and there are still standards and attribution problems, which need to be solved [15]. (3) Closed loop function: lack of effective use mechanism, online and offline medicine, makes it difficult to form a closed loop, difficult to achieve effective profit model.

### 2.2. Block Chain

The emergence of block chain has brought people unlimited imagination. Block chain electronic medical records, drug anticounterfeiting, DNA wallet, smart contract, and other technologies will completely subvert the traditional medical and health industry [16, 17]. The application of block chain and big data will be the general direction of future development, but it will take more time for the existing medical order rules and the existing information system to be fully realized. There are still many challenges at the technical and business level in block chain, such as capacity and performance problems, and security limitations.

#### 2.2.1. Logistic Regression Algorithm

In fact, logistic regression algorithm is the simplest algorithm in neural network, which involves loss function, also known as log likelihood function, and the larger the value of this function, the better [18].

(1) $$\begin{array}{c} \text{net}=\sum_{i=0}^{n}w_{i}x_{i},\\ o=\sigma \left(\text{net}\right)=\frac{1}{1+e^{-\text{net}}},\\ f\left(x\right)=\text{sigmoid}\left(w^{T}x+b\right). \end{array}$$

Now, combine the linear function with the sigmoid function. Replacing *Z* with *θ*^*T*^*x*, we get the model algorithm function:

(2) $$\begin{array}{c} h_{\theta }\left(x\right)=g\left(\theta^{T}x\right)=\frac{1}{1+e^{-\theta^{T}x}}. \end{array}$$

In the whole composite function, sigmoid is a fixed function with no parameters. So Sida is the only parameter.

RETRACTED

The purpose of constructing the loss function is that we need to have a standard under which we can find the best model that can best fit the training sample.

(1) The strategy function is
  (3) $$\begin{array}{c} {\left(h_{\theta }\left(x_{i}\right)\right)}^{y_{i}}{\left(1-h_{\theta }\left(x_{i}\right)\right)}^{1-y_{i}}. \end{array}$$
The larger the value is, the better the fitting effect of the model is.
(2) Consider the influence of samples on the model:
  (4) $$\begin{array}{c} \prod_{i=1}^{m}{\left(h_{\theta }\left(x_{i}\right)\right)}^{y_{i}}{\left(1-h_{\theta }\left(x_{i}\right)\right)}^{1-y_{i}}. \end{array}$$
For *M* samples, the larger the value of the above formula is, the better the fitting effect of the model for *M* samples is.
(3) The loss function of logistic regression classifier is constructed:
  (5) $$\begin{array}{c} L\left(\theta \right)=\prod_{i=1}^{m}{\left(h_{\theta }\left(x_{i}\right)\right)}^{y_{i}}{\left(1-h_{\theta }\left(x_{i}\right)\right)}^{1-y_{i}}. \end{array}$$

If a certain value of the harness just makes the loss function reach the maximum, then the model corresponding to the value is the best model.

The loss formula of logistic regression classifier is to find the maximum value, but it is different to find the minimum value with general loss function. In practice, logarithm *L*(*θ*) is often used:

(6) $$\begin{array}{c} l\left(\theta \right)=\log\;L\left(\theta \right)=\sum_{i=1}^{m}\left(y_{i}\log\;h_{\theta }\left(x_{i}\right)+\left(1-y_{i}\right)\log\left(1-h_{\theta }\left(x_{i}\right)\right)\right). \end{array}$$

After taking logarithm, we call it log likelihood function.

Derivation of the above formula:

(7) $$\begin{array}{c} \frac{\partial L\left(\theta \right)}{\partial \theta }=\sum_{i=1}^{n}y_{i}x_{i}-\sum_{i}^{n}\frac{e^{\theta^{T}x_{i}}}{1+e^{\theta^{T}x_{i}}}x_{i}=\sum_{i=1}^{n}\left(y_{i}-\sigma \left(\theta^{T}x_{i}\right)\right)x_{i}. \end{array}$$

Iteration weight:

(8) $$\begin{array}{c} \theta_{j}=\theta_{j}+\alpha \sum_{i=1}^{m}\left(y_{i}-h_{\theta }\left(x^{\left(i\right)}\right)\right)x^{\left(i\right)}. \end{array}$$

The iterative process is not necessarily convergent.

#### 2.2.2. Evaluation Index of Classification Algorithm

The accuracy rate can measure the ratio of the number of positive samples with correct classification to all positive samples, and the recall rate can measure the ratio of the number of positive samples with correct classification to all positive samples [19]. Let a be the correct set, and B the wrong set:

(9) $$\begin{array}{c} \text{Precision}\left(A,B\right)=\frac{\left|A\cap B\right|}{\left|A\right|},\\ \text{Recall}\left(A,B\right)=\frac{\left|A\cap B\right|}{\left|B\right|}. \end{array}$$

Coverage refers to the proportion of the number of selected samples in the sample pool.

(10) $$\begin{array}{c} \text{Accuracy}=\frac{1}{n}\sum_{i=1}^{n}1\left({\hat{y}}_{t}=y_{t}\right). \end{array}$$

Support can measure the frequency of AB occurring at the same time. If the frequency is small, the correlation of AB is small; otherwise, the correlation is strong. Confidence measures whether B will appear or its probability when A appears. If the confidence level is low, it means that the appearance of A has little to do with the appearance of B; otherwise, it means that the appearance of a has much to do with the appearance of B.

(11) $$\begin{array}{c} \text{Support}\left(A⟶B\right)=P\left(A\cup B\right),\\ \text{Confidence}\left(A⟶B\right)=P\left(B|A\right). \end{array}$$

F1 score is the harmonic average of precision rate and recall rate, which is closer to the smaller value of precision rate and recall rate.

(12) $$\begin{array}{c} F1=\frac{2\times \text{precision}\times \text{recall}}{\text{precision}+\text{recall}}. \end{array}$$

In the future, the application prospect of the combination of intelligent medicine and block chain technology is extremely broad. In the future, we will make important discoveries on intelligent medicine, artificial intelligence, medical robots, block chain technology, 3D printing technology, medical data, and biotechnology. These six technological innovations will completely change our traditional medical model [20, 21]. From the perspective of complexity and technical level, the automation of robot process is extremely accurate. From the perspective of medical accuracy, it is a perfect combination of intelligence. This development process requires the joint efforts of all personnel.

RETRACTED

### 2.3. PICC-Related Complications

PICC in Chinese means peripherally inserted central catheter. It is the use of catheter insertion, into the vein from the arm vein close to the heart, thereby reducing the drug stimulation vascular effects, to avoid direct contact with the arm vein of a drug [22].

Indications for PICC catheter insertion: (1) long-term intravenous injection is required, but the epidermal vein is not in good condition, so it is not easy to puncture successfully; (2) repeated injection of stimulants such as chemicals; (3) long-term injection of drugs such as high permeability or viscosity, high sugar, fat emulsion, and amino acids; (4) rapid injection of pressure or pressure pump; (5) repeated blood transfusion and plasma transfusion Products, platelets, etc.; (6) people who need to collect blood samples many times a day [23, 24].

The advantages of PICC are as follows: (1) if PICC is configured, the puncture point is located in the peripheral surface vein, and there will be no life-threatening complications such as blood pulmonary artery, large vessel puncture, infection, air blockage, and large-scale vasodilation. And the success rate of puncture is extremely high, and there are not too many restrictions on the action of patients [25, 26]. (2) It can relieve the pain caused by repeated venous infection. The treatment method is simple and easy to implement. It is not limited by time and place. It can be directly treated indoors [27]. (3) The material of PICC probe is special polyurethane with excellent performance and flexibility. The catheter is extremely soft and can be stored in vivo for 6 months to 1 year [28]. (4) Because the catheter can directly enter the superior vein through a large amount of blood flow, it can quickly relieve local pain, necrosis, and phlebitis, especially caused by osmotic pressure or chemotherapy [29]. In the initial stage, patients receiving catheter therapy will not suffer from major venous injury during chemotherapy, which ensures a safe channel for the successful completion of chemotherapy in the process of intravenous chemotherapy. It provides comfortable, safe, fast, and effective venous access and provides long-term intravenous nutrition support and drug support for critically ill patients and chemotherapy patients [30].  Figure 1 shows the adaptability and advantages of PICC.

## 3. Based on the Wisdom Medical Block Chain of Digestive System Malignant Tumor Patients with PICC Catheter-Related Complications and Protective Nursing Research Experiment

### 3.1. Nursing Research Subjects of PICC-Related Complications

From February 2018 to February 2019, 98 patients with digestive system malignant tumor who underwent PICC catheterization in a hospital were selected. The requirements of the experimental objects were as follows: firstly, the patients should be confirmed by the hospital; and the indicators of PICC operation should be met; thirdly, all patients have been informed and signed the informed consent, which was approved by the hospital ethics committee. Exclusion criteria: physical conditions did not meet the requirements of PICC intubation, such as liver and kidney dysfunction [31] and cardiovascular and cerebrovascular diseases.

RETRACTED

There were 57 males and 41 females, aged from 30 to 82 years, with an average of 56.2 ± 2.3 years; the catheterization time was 4 days to 5 months, with an average of 3.2 ± 0.6 months; the types of malignant tumors in digestive system: 55 cases of gastric cancer, 28 cases of colorectal cancer, and 15 cases of esophageal cancer.

### 3.2. Experimental Methods

All patients underwent PICC catheterization, 4 fr PICC catheter (Bard, USA) was selected, and appropriate local venipuncture was selected according to the specific situation of patients. There were 51 cases of basilic vein, 30 cases of median cubital vein, and 17 cases of cephalic vein. Strictly carry out aseptic operation, help patients lie flat and stretch, and puncture contralateral shoulder with head deflection. After puncture, compress with rubber band for 24 hours, and take chest X-ray to know the position of catheter end in detail. The length of catheter was 45–55 cm. After the catheter was installed, the venous catheter was used regularly, and the square position was fixed with transparent 3 M membrane. The dressing film was changed after 24 hours and once a week. Flush the catheter with an appropriate amount of salt water every day and seal the catheter under positive pressure. After 24 hours of puncture, help the patient raise the arm and elbow, and guide the patient to carry out appropriate physical activities.

During the nursing period, the PICC catheter-related complications of patients were recorded in detail, effective protective measures were taken, and the incidence of PICC catheter-related complications before and after was compared.

### 3.3. Statistical Analysis

In this paper, the statistical software spss19.0 was used. The data in this paper were expressed as *n* (%), and the chi square test was used for comparison between groups. When *P* < 0.05, the difference between representative groups was significant, with statistical significance.

Figure 2 is the technical roadmap of this experiment.

## 4. Based on Wisdom Medical Block Chain of Digestive System Malignant Tumor Patients with PICC Catheter-Related Complications and Protective Nursing Research and Analysis

PICC catheter is an important chemotherapy method for patients with digestive system cancer, which has been widely used in clinical diagnosis and treatment abroad in recent years. The application of this surgical technique can not only reduce the pain caused by repeated puncture in patients with malignant tumor, but also avoid the local necrosis directly caused by chemical drugs, but also we cannot ignore some complications. Therefore, it is extremely important to analyze the causes of PICC-related complications, refer to venous surgery and nursing technology, reduce the impact of related complications, and implement nursing countermeasures for patients.

RETRACTED

### 4.1. Factors Affecting PICC Catheter-Related Complications

Check patient baseline data in detail, and assign values after categorizing each factor; see Table 1.

The related complications of PICC were analyzed by logistic regression. Elderly patients (>60 years old), history of drug allergy, history of diabetes, more puncture times, unreasonable catheter front position, late nursing time, etc. all these were the main causes of PICC catheter complications in chemotherapy patients (*P* < 0.05). See Table 2 and Figure 3 for details.

### 4.2. Experimental Results of PICC Catheter-Related Complications and Protective Nursing Research for Patients with Digestive System Malignant Tumor Based on Smart Medical Block Chain

As shown in Table 3 and Figure 4, 50 cases of PICC-related complications occurred during chemotherapy, with a frequency of 16.7%. Among them, 16 cases (5.3%) had puncture point bleeding, and 12 cases (4.0%) had phlebitis. Catheter occlusion was found in 9 cases (3.0%), skin allergy in 8 cases (2.7%), and thrombosis in 5 cases (1.7%). Phlebitis is the most common complication after PICC in malignant tumor patients. In order to reduce the occurrence of phlebitis, it is necessary to evaluate the venous state of patients in detail, select the appropriate PICC catheter type and venipuncture site type according to the specific situation, achieve the maximum one-time success as far as possible, and reduce the mechanical venous injury caused by repeated puncture [31]. If phlebitis occurs, ice can be applied within a certain period of time, and anti-inflammatory ointment can be used to relieve the patient's symptoms.

In order to exclude the confounding effect of other variables, Cox regression model was used to analyze the factors with statistical difference in Kaplan Meier survival analysis. Taking the occurrence of PICC-related complications in tumor patients as the dependent variable, the Cox regression model was used to analyze the gender, diabetes history, patch type, maintenance mode, maintenance cycle, and white blood cell count before catheterization as the independent variables, and the time-dependent Cox regression model was used to analyze the age variables that did not meet the equal proportion risk hypothesis. Age, film type, and white blood cell count before catheterization were set as dummy variables. Cox regression analysis showed that diabetes history, maintenance cycle, and maintenance mode were the influencing factors of PICC complications during chemotherapy (*P* < 0.05). See Table 4.

RETRACTED

It can be seen from Table 5 and Figure 5 that the effect of catheter type, puncture technology, catheter tip position, maintenance factors, fixation method, and maintenance method on catheter prolapse was analyzed by chi square test. The results showed that there were significant differences in catheter tip position and fixation method (*P* < 0.05).

The so-called catheter prolapse refers to the partial or complete detachment of the catheter from the superior vein. This is mainly related to the patient's reduced compliance, excessive hand and foot activity, and unstable sweat secretion. In order to solve this situation, it is necessary to solve the following points. (1) Patients who are prone to sweating need to strengthen the observation of the catheter, disinfect the dressing that is about to fall off, and paste it again. (2) The length of the catheter left outside the body should not be too long. Ensure that the puncture point is clean and dry, and the dressing is pasted smoothly to avoid air residue. (3) In order to reduce the movement of catheter arm and strengthen health guidance, in order to avoid excessive elbow bending, it is strictly forbidden for the patient to lift or lift the weight on the side wrist.

The experimental group was better than the control group in the knowledge and compliance of PICC catheterization, *P* < 0.05, as shown in Table 6.

As can be seen from Figure 6, compared with the control group, the experimental group had less nausea and vomiting, incision infection, abdominal distension, and other related complications after PICC nursing, and the score was better than that of the control group, *P* < 0.05.

Infection is mainly local infection and systemic infection, the most common complication of PICC in patients with malignant tumor. Among them, local infection is mainly related to premature dressing change, nonstrict aseptic surgery, and imbalance of puncture skin state. The main symptoms of systemic infection are high fever, cold, and rapid heartbeat. Because PICC catheter insertion is intervention, especially in summer, it is easy to cause bacterial invasion, and the possibility of infection becomes higher. Therefore, in order to effectively avoid the occurrence of infection, strict aseptic surgery should be carried out first. Wash hands carefully before inserting the catheter, change dressings regularly, and carefully observe the redness, fever, pain, and other symptoms of patients. When the symptoms of high temperature appear, it is necessary to culture the blood bacteria in the catheter in time, take out the catheter according to the need, and select the appropriate sensitive antibiotics according to the test results.

RETRACTED

Table 7 and Figure 7 show the satisfaction of PICC control group and experimental group for nursing service after treatment. Compared with the control group, the overall satisfaction of the experimental group was higher, *P* < 0.05.

## 5. Conclusion

This paper mainly focuses on the protection and nursing of PICC catheter-related complications in patients with digestive system malignant tumor based on smart medical block chain. Based on the previous research results of PICC catheter-related complications, combined with the latest technology of smart medical block chain, this paper studies the specific situation of patients with digestive system malignant tumor. The main purpose of this study is to analyze the causes of its complications and put forward effective protective measures to reduce the incidence of PICC-related complications through protective nursing research.

The innovation of this paper lies in the following: first, the combination of qualitative analysis and quantitative analysis, full of qualitative analysis on the basis of the analysis of data; second, the combination of theoretical research and empirical research, in-depth study of smart medical block chain technology and other theoretical basis, combined with the specific situation of patients with digestive system cancer for empirical research. Third, on the basis of smart medicine, we should make full use of the protective nursing method to reduce the incidence of PICC catheter-related complications and reduce the medical pain of patients with digestive system cancer.

In general, PICC catheter-related complications mainly include phlebitis, catheter prolapse, infection, and other symptoms. Therefore, based on the causes of PICC catheter-related complications, we should carry out appropriate protective nursing before and after PICC catheterization, adopt strict bacteria-free environment for all operations, and pay close attention to the physical characteristics of patients. After successful insertion of catheter, we should continue to carry out health education and guidance for patients to avoid excessive activity or exercise, which can effectively reduce the incidence of related complications.

## Figures and Tables

**Figure 1:** Adaptability and advantages of PICC tube.

**Figure 2:** The technology roadmap of the experimental research in this paper.

**Figure 3:** Logistic regression analysis of PICC catheter-related complications in patients with digestive system malignant tumor undergoing chemotherapy.

**Figure 4:** Types of PICC-related complications during chemotherapy.

RETRACTED

**Figure 5:** Single factor analysis of catheter prolapse.

**Figure 6:** Comparison of the knowledge and compliance scores of PICC in two groups.

**Figure 7:** Comparison of nursing service satisfaction between two groups of patients with PICC in tumor chemotherapy.

**Table 1:** Factors and evaluation of complications related to PICC catheter.

Project	Code	Assignment
Gender	X1	1 = male, 2 = female
Age	X2	1 = under 40 years old, 2 = 40–59 years old, 3 = 60 years old and above
Height	X3	1 = below 160 cm, 2 = 161–170 cm, 3 = 171–180 cm, 4 = above 181
Weight	X4	1 = below 40 kg, 2 = 41–50 kg, 3 = 51–60 kg, 4 = above 60 kg
Smoking	X5	1 = yes, 2 = no
Drink	X6	1 = yes, 2 = no
History of drug allergy	X7	1 = yes, 2 = no
History of diabetes	X8	1 = yes, 2 = no
Tumor types	X9	1 = gastric cancer, 2 = colorectal cancer, 3 = esophageal cancer
Times of chemotherapy	X10	1 = 1–6 times, 2 = more than 6 times
PICC catheter site	X11	1 = basilic vein, 2 = median cubital vein, 3 = cephalic vein
Catheter factors	X12	1 = catheter size, 2 = catheter model, 3 = catheter cavity number
Catheterization technology	X13	1 = direct puncture, 2 = Seldinger technique
Puncture times	X14	1 = more than 2 times, 2 = 1 success
Position of catheter tip	X15	1 = too deep, 2 = too shallow, 3 = level 6, 7 thoracic vertebrae
Maintenance mode	X16	1 = out of hospital maintenance, 2 = inhospital maintenance
Maintenance cycle	X17	1 = less than or equal to 7 d, 2 = more than 7 d

**Table 2:** Logistic regression analysis of PICC catheter-related complications in patients with digestive system malignant tumor undergoing chemotherapy.

Project	*β* value	SE value	Wald x2 value	*P* value	OR (95%CI)
Gender	1.029	0.422	4.218	＜0.05	1.318
Age	1.388	1.225	0.664	＞0.05	4.035
Height	1.268	1.527	0.904	＞0.05	4.334
Weight	1.179	1.423	0.734	＞0.05	3.856
Smoking	1.059	1.228	0.537	＞0.05	4.736
Drink	1.468	1.628	0.883	＞0.05	3.696
History of drug allergy	1.358	0.232	6.298	＜0.05	1.438
History of diabetes	1.138	0.322	4.789	＜0.05	1.228
Tumor types	1.158	1.236	0.628	＞0.05	1.438
Times of chemotherapy	1.356	1.124	0.765	＞0.05	20.33
PICC catheter site	1.337	1.459	0.867	＞0.05	3.433
Catheter factors	1.118	0.292	6.627	＞0.05	2.456
Catheterization technology	1.389	1.358	0.984	＞0.05	3.537
Puncture times	1.015	0.292	7.425	＜0.05	2.666
Position of catheter tip	1.228	0.282	6.645	＜0.05	3.458
Maintenance mode	1.129	0.845	4.817	＜0.05	3.128
Maintenance cycle	1.239	0.572	5.598	＜0.05	2.429

**Table 3:** Types of PICC-related complications during chemotherapy.

Types of PICC-related complications	Number of cases	Percentage (%)
Bleeding at puncture site	17	5.43
Phlebitis	13	4.22
Catheter blockage	9	3.31
Allergic changes of skin	9	2.92
Thrombosis	6	1.86
Total	54	17.35

RETRACTED

**Table 4:** Cox regression model analysis of common complications of PICC in patients with malignant tumor during chemotherapy.

Project	B	SE	Wald	P	HR	95.0% CI for HR	
						Lower part	Upper part
History of diabetes	0.482	0.225	5.027	0.025	1.619	1.063	2.467
Maintenance mode	−0.643	0.212	8.423	0.004	0.536	0.342	0.822
Maintenance cycle	0.481	0.232	4.282	0.039	1.616	1.035	2.548

**Table 5:** Single factor analysis of catheter prolapse.

Influence factor	Variable	Number of respondents	Catheter prolapse group (cases/%)	Noncatheter prolapse group (cases/%)	X2 value	*P* Value
Catheter model	4F	379	32 (8.44)	347 (91.56)	0.359	0.654
	5F	78	5 (6.41)	73 (93.59)		

Number of lumens	Single chamber	387	32 (8.27)	355 (91.73)	0.101	0.819
	Double cavity	70	5 (7.14)	65 (92.86)		

Catheterization technology	Direct puncture	39	2 (5.13)	37 (94.87)	0.163	0.687
	seldinger	418	35 (8.37)	383 (91.63)		

Puncture times	Once	382	31 (8.12)	351 (91.88)	0.001	1.000
	Greater than or equal to twice	75	6 (8)	69 (92)		

Venipuncture	Basilic vein	399	31 (7.77)	368 (92.23)	1.464	0.555
	Median cubital	39	5 (12.85)	34 (87.18)		
	Cephalic vein	19	1 (5.26)	18 (94.74)		

**Table 6:** Comparison of the knowledge and compliance scores of PICC in two groups.

Group	Number of cases	Mastery of PICC knowledge	Catheter compliance score
Control group	45	85.45±2.11	82.04±3.13
Experience group	45	95.24±3.24	96.34±3.28
t	—	8.222	9.121
P	—	*P* ≤ 0.001	*P* ≤ 0.001

**Table 7:** Comparison of nursing service satisfaction between two groups of patients with PICC in tumor chemotherapy.

Group	Number of cases	Satisfied	Quite satisfied	Dissatisfied	Satisfaction
Control group	45	21	15	9	36 (80.00)
Experience group	45	36	9	0	45 (100.00)
X2	—	—	—	—	10.00
P	—	—	—	—	0.0016

## Data Availability

No data were used to support this study.
